# Meta-Analysis of Knee Joint Function Recovery after Anterior Cruciate Ligament Reconstruction by Accelerated Rehabilitation Surgery

This article has been retracted.

**DOI:** 10.1155/2022/5085143

**Published:** 2022-06-29

**Authors:** Junxiang Xu, Minzhe Zheng, Zongxian Feng, Lingxiao Pan, Zhaoxiang Peng

**Affiliations:** Orthopedics department Ningbo Medical Center Lihuili Hospital, Ningbo 315000, China

## Abstract

**Objective:**

This investigation was undertaken to systematically assess the impact of increasingly rapid recovery treatment on the functional status of the knee following anterior cruciate ligament restructuring.

**Methods:**

Computer search from the establishment of the database to March 2022 in China Knowledge Network Database (CNKI), PubMed, EMBASE, ScienceDirect, CochraneLibrary, China VIP Database, Wanfang Database, and China Biomedical Literature Database (CBM). The control group was given only traditional rehabilitation training, and the observation group was treated with perioperative accelerated rehabilitation surgery intervention randomized controlled trial (RCT). Data for all included studies were extracted by two independent researchers, and the risk of bias for the quality of each included study was assessed by the Cochrane Handbook 5.1.0 criteria. Meta-analysis of the collected data by using RevMan5.4 statistical software.

**Results:**

A total of 593 articles were retrieved from the computer database and 8 RCT articles with a total of 636 samples were finally included for meta-analysis. According to the Jadad scale, the RCT score of 8 articles was ≥4 points. Meta-analysis was performed on the postoperative VAS scores of the ERAS group and the traditional rehabilitation group, and the heterogeneity test showed Chi^2^ = 288.60, d*f* = 5, *P* < 0.00001, and *I*^2^ = 99%. There was a statistically significant difference in the postoperative VAS scale between the intervention and the traditional rehabilitation model (*P* < 0.05). Eight articles reported the effect of accelerated rehabilitation surgery on the recovery of knee joint motion after ACL rehabilitation. After meta-analysis, the heterogeneity test showed Chi^2^ = 314.98, d*f* = 7, *P* < 0.00001, and *I*^2^ = 98%, and it can be concluded from the analysis that, compared with the traditional rehabilitation model, the enhanced rehabilitation surgery has an effect on the joint function after anterior cruciate ligament reconstruction. The improvement effect was more significant, and the difference was statistically significant (*P* < 0.05). Four articles reported the effect of enhanced recovery after surgery intervention on the range of motion of the knee joint of patients, the heterogeneity test showed Chi^2^ = 117.52, d*f* = 2, *P* < 0.00001, and *I*^2^ = 98%, through analysis, and compared with the traditional rehabilitation model and the enhanced recovery. The effect of surgery on the range of motion of the knee joint after ACL reconstruction was more significant, and the difference was statistically significant (*P* < 0.05). The effect of enhanced recovery after surgery and traditional rehabilitation mode on the incidence of postoperative adverse reactions in patients undergoing ACL reoperation was analyzed. The results of heterogeneity test showed that Chi^2^ = 1.59, d*f* = 2, *P*=0.66 > 0.05, and *I*^2^ = 98%, and the analysis showed that, compared with the traditional rehabilitation mode, enhanced rehabilitation surgery can significantly reduce the risk of adverse reactions after anterior cruciate ligament reconstruction (*P* < 0.05). An inverted funnel plot was used to analyze publication bias in studies with quality of life as an outcome measure. The results showed that Egger's test *P*=0.0005 < 0.001 suggesting that there may be a certain degree of publication bias.

**Conclusion:**

The existing research evidence shows that accelerating the reconstruction of anterior cruciate ligament can effectively promote the recovery of knee joint function, reduce the pain of patients, and reduce postoperative complications. However, more research is needed to further verify this.

## 1. Introduction

The knee joint anterior cruciate ligament (ACL) is one of the crucial structures to keep the knee joint stable. Rupture can lead to anterior instability and further cause knee joint subsidiary damage [1–3]. The anatomical basis, tissue structure, and biomechanical function of ACL, as well as regional economic and social factors, determine the epidemiological characteristics of ACL. ACL injury is different from other types of knee joint diseases. The particularity of ACL injury has different distribution of injured patients, and the injury mechanism of ACL also has its unique performance. According to the report, the overall incidence of former cross patients in the United States is 100/300,000, while the prevalence rate of people engaged in special sports, such as football or basketball, is as high as 60/100000, and that of skiers is 70/100,000, which is significantly higher than that of the general population [4]. And, because the knee ligament relaxation of female is higher than that of male, the muscle strength of posterior group of thigh is worse, and the diameter of ACL is smaller, so the incidence of ACL injury in female is significantly higher than that in male. At the same time, sports injury is the main cause of ACL injury. Some steering movements require higher stability of the knee joint, while producing greater traction and torsion load; sports enthusiasts often ignore the practice of muscle strength when they focus on their favorite sports, and the low level of physical quality makes the knee joint lack of reliable muscle protection during exercise, which increases the risk of injury of knee joint ACL and other stable structures. At present, arthroscopy-assisted ACL reconstruction has been very mature, and the basic research and clinical research on ACL injury and treatment at home and abroad have been very extensive and in-depth, mainly focused on the anatomical reconstruction of ligament, biomechanical reconstruction, tendon healing, renewal of fixation methods and fixation materials, durability of graft, arthroscopic minimally invasive reconstruction, postoperative rehabilitation, research and development of advanced surgical equipment, etc.

The stiffness of knee joint after ACL damage is a hot topic studied at home and abroad for many years. The postoperative recovery of knee joint function is generally poor, and this problem needs to be seriously studied and solved. In addition, the anatomical and histological features of the ACL determine its poor blood supply [5]. Therefore, after the rupture of the anterior cruciate ligament, conservative treatment cannot restore the original state. The functional instability of the affected limb cannot be corrected by nonoperative treatment [6–8] and cannot meet the needs of patients. However, with further research, most experts believe that early surgical reconstruction is needed after ACL injury, which can regain the anterior knee joint stabilization and correct rotation and prevent the further aggravation of intra-articular secondary injury. This is of great significance to the management of complications, the protection of meniscus, the protection of articular cartilage, and the protection of other ligaments in the joint.

With the progress of arthroscopic surgery, arthroscopic ACL reconstruction has become a routine treatment for ACL injury and multiple ligament injuries of the knee joint [9]. However, a series of symptoms represented by the limitation of limb movement after ACL reconstruction is a great obstacle to the recovery of limb function after the operation. Miao Shuai et al. [10] proposed that the incidence of joint stiffness and the limitation of limb movement after ACL reconstruction after ACL injury for 3 or more weeks were lower. However, a study by Guo et al. [11] and Lin et al. did not find any great differences in the incidence of joint adhesion between early and late reconstruction of ACL injury [11, 12].

The current literature [11, 13] has proved that accelerating rehabilitation surgery can promote the cases' knee joint functional recovery after ACL restructure, but the study has not been randomly assigned, and the sample size is small and lack of credibility. Therefore, through meta analysis, this study quantitatively synthesized the published randomized controlled trials (RCT), expanded the sample size, increased the statistical efficiency and the accuracy of estimated effect values, and enhanced the reliability and objectivity of the results [13]. In order to provide evidence-based evidence for postoperative rehabilitation of patients with knee anterior cruciate ligament injury.

## 2. Research Contents and Methods

### 2.1. The Sources and Retrieval Methods of Documents

Computer search was carried out from the establishment of the database to March 2022 in China Knowledge Network Database (CNKI), PubMed, EMBASE, ScienceDirect, CochraneLibrary, ChinaVIPDatabase, Wanfang Database, and China Biomedical Literature Database (CBM). The control group was given traditional rehabilitation training only, while the observation group was treated with accelerated rehabilitation surgery intervention (RCT). Literature retrieval was conducted in the way of free words and subject words, with the key words of accelerated rehabilitation surgery, nursing intervention, anterior cruciate ligament reconstruction, knee joint function, and so on.

### 2.2. Literature Inclusion Criteria and Exclusion Criteria

#### 2.2.1. Literature Inclusion Criteria

1. Type of study: all domestic patients after ACL reoperation received a randomized control test of accelerated rehabilitation surgery and traditional rehabilitation intervention (RCT). The language was limited to Chinese.
2. Participants: CT, MRI, and other imaging methods were used to confirm the diagnosis of anterior cruciate ligament injury.
3. Intervention: control patients accepted rehabilitation training and experimental patients accepted accelerated rehabilitation surgery. The main results are as follows: (1) the mode of operation: anterior cruciate ligament reconstruction. (2) Intervention: the control group was given only traditional rehabilitation training, and the study group received accelerated rehabilitation surgery during the perioperative period. (3) Outcome indicators: perioperative indicators (length of stay, postoperative complications, serum factor levels, etc.), quality of life score, VAS score, joint function score, and quality of life score.

#### 2.2.2. Literature Exclusion Criteria

The literature exclusion criteria are as follows:

(1) It is not a randomized controlled study; (2) the data report is incomplete, and the data cannot be used; (3) repeat the research content and take the latest research; (4) the expression of the research index is not clear.

### 2.3. Quality Evaluation and Data Extraction

1. Quality evaluation: the qualities of the enrolled literature were assessed by the Jadad scale, which was evaluated according to random, blind method, and loss of follow-up/withdrawal. 0–5 points were used to count. When the literature quality is less than 2 points, it is lower, and when it is ≥3 points, it is higher. The specific evaluation is as follows: (1) random: (1) 2 points: “random distribution” is mentioned in the literature and described in detail and correctly. (2) 1 score: “random distribution” is only mentioned in the literature but not explained. (3) 0: the random allocation method/random allocation/pseudorandom allocation was not mentioned in the literature. (2) Blind method: (1) 2 points: the “double-blind” method is used in the literature, and the specific process is described correctly. (2) 1: the “double-blind” method is not specifically described in the literature. (3) 0: no “double-blind” method/method error. (3) withdrawal/loss of follow-up: (1) 1: the number and reasons of withdrawal and loss of follow-up are described in detail in the literature. (2) 0: it is not mentioned in the literature.
2. Data extraction: data for all included studies were extracted by two independent researchers, and the risk of bias for the quality of each included study was assessed by the Cochrane Handbook 5.1.0 criteria. When the two people had differences, they reached an agreement through consultation. It includes study author, publication time, sample size, treatment method, and curative effect evaluation method.

### 2.4. Statistical Processing

RevMan5 software originated from the Cochrane Collaboration Network for Meta Analysis. The mean and standard deviation of the net change difference of serum albumin, prealbumin, and hemoglobin in the experiment and the control cohorts were input into RevMan5 for analysis. Because the index is a continuous variable, the weighted mean difference (WMD) is used as the effect scale, and 95% confidence interval is selected. First, the *X*^2^ test is used to determine whether there is heterogeneity between the studies. If *P* > 0.05 and *I*^2^ <50%, it is considered that the included study is homogeneous, and the modified impact model can be collected for meta-analysis; if *P* < 0.05 and *I*^2^ ≥50%, when judging the homogeneity of the included study, the combined effect is needed and then choose the random effect model; if *P* < 0.05 and the source of heterogeneity could not be judged, meta analysis was not performed, and descriptive analysis was used.

## 3. Results and Analysis

### 3.1. Literature Search Results and Basic Information of Included Literature

593 articles were retrieved through computer database retrieval, 281 articles were obtained after excluding duplicate studies, 136 articles were obtained through preliminary reading of the titles and abstracts of the articles, irrelevant studies, reviews, case reports, and uncontrolled articles were excluded, and 35 articles were initially included, and then the full text of the literature was carefully read, 27 literature with incomplete data and no primary outcome indicators were excluded, and 8 RCTs were finally included with overall 636 cases for meta analysis. The general aspects of the collected publications are displayed in Table 1.

### 3.2. Evaluation of the Quality of the Methodology Included in the Literature

Eight RCT articles included in this meta-analysis reported the baseline of patients, of which five RCT were randomized by random number table, and the other three articles did not mention the specific method of random grouping. Among them, 7 studies all gave detailed intervention measures, and 3 studies did not specify the follow-up time. The number and reasons of blind method and loss of follow-up or withdrawal were not described in detail in eight RCT articles. According to the Jadad scale, we can see that eight articles have RCT scores ≥4. The results are shown in Table 2. The results of the literature quality evaluation showed that five articles [12, 15–18] were of low risk and three [19–21] were of medium risk. The studies that were rated as medium-risk mainly showed distribution hidden bias and report bias. Risk bias is shown in Figure 1.

### 3.3. Meta Analysis Result

#### 3.3.1. VAS Scoring

Through the meta-analysis postoperative VAS scores of 636 samples from the 8 ERAS groups compared with the traditional rehabilitation group in the RCT study, the postoperative VSA scores were revealed in the overall enrolled six articles. The heterogeneity test showed that Chi^2^ = 288.60, d*f* = 5, *P* < 0.00001, and *I*^2^ = 99%, indicating that there was heterogeneity among the included research data. The postoperative VAS scores of patients after ACL reconstruction using enhanced recovery surgery intervention were significantly different from those of the traditional rehabilitation model (*P* < 0.05). The results are shown in Figure 2.

#### 3.3.2. Lysholm Scoring

The effect of accelerated rehabilitation surgery on patients' knee joint functional after ACL reconstruction was reported in 8 literature studies. Meta analysis with random effect model showed that Chi^2^ = 314.98, d*f* = 7, *P* < 0.00001, and *I*^2^ = 98%, indicating that there was heterogeneity among the included research data. Compared with the traditional rehabilitation model, accelerated rehabilitation surgery has a more significant effect on the joint functional improvement after ACL reconstruction (*P* < 0.05). The results showed that the effect of accelerated rehabilitation surgery on the joint function of patients after anterior cruciate ligament reconstruction was significantly better than that of traditional rehabilitation mode. The results are shown in Figure 3.

#### 3.3.3. Range of Motion of Knee Joint

Among the eight articles included in the study, four reported the effect of accelerated rehabilitation surgical intervention on the range of motion of patients' knee joints. The heterogeneity test displayed Chi^2^ = 117.52, d*f* = 2, *P* < 0.00001, and *I*^2^ = 98%, indicating that there is heterogeneity among the included research data. Compared with the traditional rehabilitation model, accelerated rehabilitation surgery has a more significant effect on the scope of knee joint movements after ACL reconstruction (*P* < 0.05). The results are shown in Figure 4.

#### 3.3.4. Complication

Four studies with extractable adverse reactions were analyzed by meta-analysis. The main adverse reactions included joint cavity effusion, joint cavity hemorrhage, infection, adhesive arthritis, and nerve injury, and no serious adverse reactions were reported. The effects of accelerated rehabilitation surgery and traditional rehabilitation model on the incidence of postoperative adverse reactions in patients with anterior cruciate ligament reconstruction were compared with those in these four studies. The results of heterogeneity test showed that Chi^2^ = 1.59, d*f* = 2, *P*=0.66 > 0.05, and *I*^2^ = 98%, indicating that there was no obvious heterogeneity among the included data, and the combined effect of WMD was analyzed by the fixed effect model. The combined effect size WMD test is *Z* = 4.31 (*P* < 0.00001). According to the analysis results, it can be considered that compared with the traditional rehabilitation mode, the use of enhanced recovery surgery can significantly reduce the number of patients after ACL rebuilding. The risk of adverse reactions was greatly distinct (*P* < 0.05). The results are shown in Figure 5.

#### 3.3.5. Publication Bias Analysis

An inverted funnel plot was used to analyze the publication bias of studies with quality of life as the outcome indicator. The results are shown in Figure 6. The results showed that the graphs were not completely symmetrical, and the Egger's test showed *P*=0.0005 < 0.001, suggesting that there may be a certain degree of publication bias.

## 4. Analysis and Discussion

Anterior cruciate ligament (ACL) is of remarkable meaningful for keeping the knee joint anterior stability and controlling the knee joint rotation. It is divided into the anterior medial bundle and the posterior lateral bundle. Its special anatomical characteristics determine that the tension of the two bundles of the knee joint is different during movement and changes accordingly with the extension and flexion of the knee joint. The anatomical position of the anteromedial ligament of the tibia determines its function, which mainly restricts the forward movement of the tibia and prevents the tibia from being damaged during movement. The anatomical position of the posterolateral bundle determines its function, which mainly restricts the backward movement of the knee joint. Therefore, the mechanism of its stability is to prevent the tibia from slipping forward in the joint during knee flexion, to prevent knee joint hyperextension during knee extension, and to actively control knee joint rotation and valgus under different knee flexion angles. According to Noyes's previous biomechanical tests, ACL assumed most of the antagonistic forces of the anterior drawer test when the knee was flexion 90° and the tibia was in a neutral position. ACL damage can cause knee joint instability to varying degrees and influence the knee joint functional activities, and the ACL rupture changes the stress form of meniscus and intra-articular cartilage itself. Therefore, to restore knee joint function to normal activity level as far as possible, most doctors advocate that ligament reconstruction should be actively carried out for patients with ACL [22]. Accelerating rehabilitation program is a more active rehabilitation strategy. It can reduce joint adhesion and increase joint range of motion in order to restore the intact structure and stabilization of the injured knee joint and eliminate the knee joint complications under conservative treatment [23].

With the renewal of the concept of knee rehabilitation, the recovery level of postoperative motor ability has been greatly improved in the past 30 years. Accelerated rehabilitation surgery (ERAS) is a perioperative management method based on evidence-based medicine, which can reduce surgical trauma, reduce physical and psychological trauma stress, accelerate patient recovery, shorten hospital stay, and reduce hospitalization costs [24]. At the same time, it is a new type of perioperative medical cooperation project with surgery, anesthesiology, nursing, rehabilitation therapy, and so on. It includes reasonable perioperative management, such as fast-track anesthesia, minimally invasive surgery, best analgesic techniques, early postoperative feeding, and early getting out of bed. ERAS takes patient safety as the premise and rapid recovery as the goal, integrates various perioperative medical and nursing measures, and allows patients to pass through the perioperative period “safely and quickly.” There was no significant difference between the accelerated rehabilitation program and the conventional rehabilitation program in joint range of motion, muscle strength, and stability, but the rehabilitation time was significantly longer than that of the conventional rehabilitation program [25, 26]. Early out-of-bed exercise and functional training can improve the symptoms of limited joint movement after ACL reconstruction, mostly in cases where knee joint movement is strictly restricted after the operation. Joint range of motion and weight-bearing activity aggravate lower limb muscle atrophy to some extent and promote the recovery of knee joint function [27]. The concept of early active rehabilitation is to carry out functional exercise of rehabilitation nature as soon as possible, which can help shorten the time for functional recovery of the knee joint and help improve the effect of knee joint surgery [14, 28]. Although early studies have shown that accelerated rehabilitation programs do not adversely affect the prognosis of patients like conventional rehabilitation programs [29]. Most rehabilitation programs for ACL reconstruction take 6 months as a cycle.

At present, there is still a lack of high-level evidence-based evidence about the value of accelerated rehabilitation surgery [30]. Based on this, through meta-analysis, this paper systematically evaluates the effect of accelerated rehabilitation surgery on knee joint functional recovery after ACL reconstruction, so as to provide evidence-based reference for clinical treatment. Totally, eight RCT studies with overall 636 patients were enrolled in this investigation. Six of them scored postoperative VAS. A meta-analysis was performed on the postoperative VSA scores in these 6 studies. There was a large discrepancy in the following surgery VAS score between patients after enhanced rehabilitation surgery intervention for anterior cruciate ligament reconstruction and the traditional rehabilitation model (*P* < 0.05). Eight reported the effect of accelerated rehabilitation surgery on the knee joint functional restore after ACL operation. The effect of accelerated rehabilitation surgery on joint function of patients after anterior cruciate ligament reconstruction was more significant than that of traditional rehabilitation model (*P* < 0.05). Of the eight studies included in the study, four reported the effect of enhanced recovery after surgery intervention on the range of motion of the knee joint of patients. According to the different intervention measures, it was found that compared with the traditional rehabilitation model, upon the use of enhanced recovery after surgery, the improvement effect on the scope of knee joint motion in patients after ACL reoperation was more significant (*P* < 0.05). Four studies on the number of extractable ADR cases were analyzed by meta-analysis, and the occurrence of ADR was reported in all 4 studies. The main adverse reactions included articular effusion, articular hemorrhage, infection, adhesive arthritis, and nerve injury. No serious adverse reactions were reported. Among the eight articles included, four articles compared the effects of accelerated rehabilitation surgery and traditional rehabilitation model on the incidence of postoperative adverse reactions in patients with anterior cruciate ligament reconstruction. Accelerated rehabilitation surgery can significantly reduce the risk of adverse reactions in patients after ACL reoperation (*P* < 0.05). Among the studies included in this analysis, some studies have been observed for a short time, and the recovery of joint function is a long-term and chronic process. The effect of accelerated rehabilitation surgery on the knee joint functional improvement after ACL reoperation may be more significant after long-term follow-up, but the actual effect still needs a lot of studies to confirm.

## Figures and Tables

**Figure 1:** Risk of bias assessment of included studies.

**Figure 2:** Forest plot of the impacts of accelerated rehabilitation surgery on the VAS scale.

**Figure 3:** Forest plot of the joint function recovery.

**Figure 4:** Forest plot of effect of accelerated rehabilitation surgery on the range of motion of knee joint.

**Figure 5:** Forest plot of impacts of accelerated rehabilitation surgery on postoperative complications.

**Figure 6:** Inverted funnel plot of the impact of accelerated restore operation on the life quality of patients.

**Table 1:** Basic information of included studies.

Included literature	Year of publication	*N* (T/C)	Study group interventions	Control group interventions	Follow-up time	Observation indicator
Guo et al. [13]	2022	30/30	Accelerated rehabilitation surgery	Traditional rehabilitation	12 months	①②④
Lin et al. [12]	2020	61/57	Accelerated rehabilitation surgery	Traditional rehabilitation	Unknown	①②③
Qin et al. [14]	2020	43/42	Accelerated rehabilitation surgery	Traditional rehabilitation	6 months	①②④
Zhang et al. [15]	2020	44/44	Accelerated rehabilitation surgery	Traditional rehabilitation	Unknown	②④
Xu et al. [16]	2020	37/38	Accelerated rehabilitation surgery	Traditional rehabilitation	3 months	①②③④
Zhao et al. [17]	2021	37/38	Accelerated rehabilitation surgery	Traditional rehabilitation	Unknown	①②
Ge et al. [18]	2021	50/25	Accelerated rehabilitation surgery	Traditional rehabilitation	2 weeks after operation	①②
Yan et al. [19]	2020	30/30	Accelerated rehabilitation surgery	Traditional rehabilitation	On the day of discharge	1 ②

Note: ① VAS score; ② knee joint function score; ③ postoperative complication; ④ range of motion of joint.

**Table 2:** Results of methodological quality evaluation.

First author and year of publication	Random	Randomized hiding	Blind method	Withdrawal and dropouts	Total	Quality grade
Guo et al. [13]	2	1	1	1	5	High
Lin et al. [12]	1	1	1	1	4	High
Qin et al. [14]	2	1	1	1	5	High
Zhang et al. [15]	2	1	1	1	5	High
Xu et al. [16]	2	1	1	1	5	High
Zhao et al. [17]	1	1	1	1	4	High
Ge et al. [18]	1	1	1	1	4	High
Yan et al. [19]	2	1	1	1	5	High

## Data Availability

No data were used to support this study.

## References

[1] Mistry H., Metcalfe A., Colquitt J. (2019). Autograft or allograft for reconstruction of anterior cruciate ligament: a health economics perspective. *Knee Surgery, Sports Traumatology, Arthroscopy*.

[2] Smith P. A., Thomas D. M., Pomajzl R. J., Bley J. A., Pfeiffer F. M., Cook J. L. (2019). A biomechanical study of the role of the anterolateral ligament and the deep iliotibial band for control of a simulated pivot shift with comparison of minimally invasive extra-articular anterolateral tendon graft reconstruction versus modified lemaire reconstruction after anterior cruciate ligament reconstruction. *Arthroscopy: The Journal of Arthroscopic & Related Surgery*.

[3] Riaz O., Aqil A., Mannan A. (2018). Quadriceps tendon-bone or patellar tendon-bone autografts when reconstructing the anterior cruciate ligament: a meta-analysis. *Clinical Journal of Sport Medicine*.

[4] Jin C., Song E. K., Jin Q. H., Lee N. H., Seon J. K. (2018). Outcomes of simultaneous high tibial osteotomy and anterior cruciate ligament reconstruction in anterior cruciate ligament deficient knee with osteoarthritis. *BMC Musculoskeletal Disorders*.

[5] Trung D. T., Manh S. L., Nguyen Thanh L., Chu Dinh T., Chu Dinh T. (2019). Preliminary result of arthroscopic anterior cruciate ligament reconstruction using anterior half of peroneus longus tendon autograft. *Open Access Macedonian Journal of Medical Sciences*.

[6] Rusanov A., Kravchuk L., Rusanova O., vitaly Z., olga S. (2018). Physical Rehabilitation of patients who underwent the reconstruction of anterior cruciate ligament with arthroscopic surgical interventions. *Journal of Physical Education and Sport*.

[7] Gu X., Wei X. (2020). A meta analysis of early versus delayed reconstruction of anterior cruciate ligament injuries in adolescents is associated with the risks of meniscus and articular cartilage injury. *Osteoarthritis and Cartilage*.

[8] Yang L., Zou C., Mi Y., Wang Z. (2021). All-inside reconstruction of anterior cruciate ligament with single-bundle autogenous peroneal longus tendon. *Orthopaedic Journal of Sports Medicine*.

[9] Gupta R., Gupta A. (2021). A recent follow-up study on reconstruction of anterior cruciate ligament by arthroscopic free hamstring transplantation and retaining inserted hamstring transplantation. *Journal of Contemporary Medical Practice*.

[10] (2019). Accelerated rehabilitation programme after arthroscopic reconstruction of anterior cruciate ligament. *Eur J Ther*.

[11] Guo B., du J., Wang L. (2022). Effect of accelerated rehabilitation surgery on function after anterior cruciate ligament reconstruction of knee joint. *Chinese contemporary medicine*.

[12] Lin L., Xiong Y., Qin Q. (2020). Effect of accelerated rehabilitation surgical nursing on the function of anterior cruciate ligament reconstruction of knee joint. *Chinese medical science*.

[13] Karakoc Z. B., Colak T. K., Zubeyir S. A. R. I., Mine G .P (2019). The effect of virtual rehabilitation added to an accelerated rehabilitation program after anterior cruciate ligament reconstruction: a randomized controlled trial. *Clinical and Experimental Health Sciences*.

[14] Qin A., Lei D., Huang Q. (2020). Effect of rapid rehabilitation on knee joint function after arthroscopic anterior cruciate ligament reconstruction. *Medical theory and practice*.

[15] Zhang X. (2020). Effect of rapid rehabilitation concept on knee joint function and complications after arthroscopic anterior cruciate ligament reconstruction. *Medical dietotherapy and health*.

[16] Xu X., Yang L. (2020). Effect of rapid rehabilitation surgery in arthroscopic anterior cruciate ligament reconstruction. *Clinical medical research and practice*.

[17] Zhao W., Sun J., Wang Y. (2021). Effect of rapid rehabilitation and traditional rehabilitation on postoperative functional recovery in military patients with anterior cruciate ligament reconstruction. *Armed police medicine*.

[18] Ge R., Lu J., Zhang C. (2021). Application effect of rapid rehabilitation surgery in anterior cruciate ligament reconstruction. *Journal of practical Orthopaedics*.

[19] Yan D., Xu Y., Gu S. (2020). Observation on the effect of rapid rehabilitation nursing after anterior cruciate ligament reconstruction. *Journal of Changchun University of traditional Chinese Medicine*.

[20] Sun K., Chen L., Mai Y. (2021). Clinical application of enhanced recovery after surgery in the perioperative period of anterior cruciate ligament reconstruction. *Chinese Journal of Tissue Engineering Research*.

[21] Karakoc Z. B., Colak T. K., Sari Z., Gülden P. M. (2019). The effect of virtual rehabilitation added to an accelerated rehabilitation program after anterior cruciate ligament reconstruction: a randomized controlled trial. *Clinical and Experimental Health Sciences*.

[22] Liang Z., Ding J., Chen B. (2021). Research progress of ulnar collateral ligament reconstruction in the treatment of ulnar collateral ligament injury in over-top throwing athletes [J]. *Chinese Journal of Orthopaedic Trauma*.

[23] Shuai M., Li S., Wu Z., Wang H., Li M. (2021). The clinical efficacy and risk factors after revision and reconstruction of anterior cruciate ligament. *Journal of healthcare engineering*.

[24] Luo Y., Zhang C., Wang J. (2021). Clinical translation and challenges of biodegradable magnesium-based interference screws in ACL reconstruction. *Bioactive Materials*.

[25] Huang S., Xie Y., Huang Z. Preoperative predictors of prolonged hospital stay in accelerated rehabilitation for patients undergoing orthopedic surgery. *Bioinorganic Chemistry and Applications*.

[26] Lieber A. C., Steinhaus M. E., Liu J. N., Hurwit D., Chiaia T., Strickland S. M. (2019). Quality and variability of online available physical therapy protocols from academic orthopaedic surgery programs for medial patellofemoral ligament reconstruction[J]. *Orthopaedic Journal of Sports Medicine*.

[27] Gerritsen L. M., van der Lelij T. J. N., van Schie P. (2022). Higher healing rate after meniscal repair with concomitant ACL reconstruction for tears located in vascular zone 1 compared to zone 2: a systematic review and meta-analysis. *Knee Surgery, Sports Traumatology, Arthroscopy*.

[28] Zhao J. (2020). Anatomical single-bundle transtibial anterior cruciate ligament reconstruction. *Arthroscopy techniques*.

[29] Foissey C., Thaunat M., Bondoux L., Sonnery-Cottet B., Fayard J. M. (2021). Self-rehabilitation guided by a mobile application after anterior cruciate ligament reconstruction leads to improved early motion and less pain. *Arthroscopy, sports medicine, and rehabilitation*.

[30] Zhao J., Qiu J., Chen J., Xu J. (2020). Combined double-bundle anterior cruciate ligament reconstruction and anterior cruciate ligament-mimicking anterolateral structure reconstruction. *Arthroscopy techniques*.

